The article "A New Approach for Target Capability Assessment and Selection in Complex Situations" was published in 2022. Journal: Comput Intell Neurosci.

# A New Approach for Target Capability Assessment and Selection in Complex Situations

**DOI:** 10.1155/2022/3146683

**Published:** 2022-08-31

**Authors:** Yuan Wang, Jun Liang, Shicheng Wang

**Affiliations:** Department of Control and Engineering, Research Institute of High Technology, Xi'an 710025, China

## Abstract

In modern information warfare, medium and long-range weapons with high strike precision are often used to ensure stable, accurate, and ruthless conditions. However, the target system often has multiple target units and which target units to specifically attack becomes the primary issue. This study constructs a target combat system network based on the complex network theory and maximum entropy principle, establishes a key target selection model based on this network, and then determines the use of medium and long-range weapons to strike the key target unit in the enemy combat system network. The key target selection model consists of four parts. The first is a value model of the node itself constructed by comprehensively considering the relationship between the target and the war, the importance of the target in the system, and the threat of the target. The second is a node network value model based on the potential field theory. The third is to construct a cascading failure model of the target system through the definition of triples (results of strike action, target unit status, and failure influence relationship between target units). Fourth, with the optimal cost-effectiveness ratio as the objective function, the evaluation criterion function model is established. Case scenarios and simulation experiments illustrate the rationality and effectiveness of the method which can provide effective solutions for commanders to select key targets.

## 1. Introduction

The complex network is an important tool used to describe the real social network. In application, the system is usually abstracted into a network, and a directed graph is used to describe it, and then, its attributes are mathematically modeled and analyzed. Watts and Strogatz [1] proposed a small-world network model, which can be regarded as the pioneering work of complex network models. As a result, the complex network has attracted the attention of many scientific researchers and has become a hot research topic. It has now been applied in various fields. Hu et al. [2] proposed to establish a connection between complex networks and patients with concurrent diseases, which promotes the development of targeted treatment programs. Zhao et al. [3] studied the time synchronization mechanism of multilink complex networks based on the concept of drive response and infinite time stability theory. Yafei [4] proposed a health system evaluation construction method based on system dynamics and complex networks, which improves the rationality of the health policy evaluation system index planning. Lu et al. [5] put forward a potential evaluation model of the accessibility index of the public bicycle complex network on the basis of analyzing the characteristics of complex network topology, which provides a theoretical basis for the optimization of the public bicycle system. Nevertheless, complex networks have not been well utilized in the military combat system. Modern warfare is often an informationized war between combat systems and systems, which involve multiple platforms, such as combat, support, and reconnaissance, and there are different relationships between these platforms. Such wars are composed of complex and huge networks. Ruan et al. [6] applied the idea of complex networks to air defence weapon systems and determined the order of target strikes through the measurement of node degree and node betweenness. Although the relationship between directly adjacent nodes is considered in this paper, there is no research on the influence of indirect adjacent nodes. Yan and Zia [7] used complex network theory to build an antilanding deployment network model, and through the value evaluation of nodes, it provides a basis for selecting targets for airborne operations. Although the studies also considers the network value of nodes and the role of nodes in ensuring the normal operation of the entire network, the interaction between nodes and the role of alternate nodes are not added.

Due to the complex and huge network of the enemy's combat system, the number of our strike weapons is unlikely to be able to strike all of the enemy's targets. Therefore, the target should be the key nodes and key targets in the enemy's combat system, which can weaken or destroy the enemy's combat capability at a minimum cost. At present, the main research ideas for the selection of key targets in the target system are using the analytic hierarchy process, influence network, influence diagram, fuzzy clustering method, approach to ideal solution method, gray theory, Bayesian network, fault tree, and graph theory to analyze the system model and then combine other statistical methods such as ranking to determine the priority of goals or actions. Zhang and Xiao [8] comprehensively considered the effective range, command and control capabilities, penetration capabilities, and target characteristics of shipborne weapons. According to the weapon combat model, the analytic hierarchy process is used to obtain the capabilities of the weapon. And then which kind of weapon equipped with the ability required can be found by ranking. The analytic hierarchy process can achieve good results when considering fewer factors, but for a complex network such as a combat system, the workload is very large and it is also very difficult to consider the integrity of factors. Falzon and Pousi [9, 10], respectively, used probability networks such as Bayesian networks, influence networks, and influence diagrams to study complex target systems, but these methods all need to input a large number of conditional probabilities and have poor reusability of network topology. Du et al. [11] used fuzzy cluster analysis to sort the main shooting areas to select targets to be hit. However, the target regional system established by it lacks correlation and only considers the state of ability within a single region. Wu and He [12] modeled the benefits of strike targets from the degree of relevance, system importance, threat level, strike cost, and strike risk and proposed a method based on data envelopment analysis-approximate ideal solution sorting method to rank targets, thus selecting the target that maximizes the effectiveness of combat. For a single target to be hit, the factors considered in the study are more comprehensive, but it lacks the intuition brought by the complex network and cannot consider the problem of cascading failure. Han et al. [13] considered a variety of factors that affect the decision of a single target and then used a combination of the analytic hierarchy process and gray correlation method to sort the targets, so as to determine the priority of hitting the target. However, the object of the study is the single target rather than the multitarget system, and the generalized indicators given cannot include the relevance and indirect relevance of network definition factors in the study. Lei et al. [14] used an object-oriented Bayesian network to analyze the topological structure of the failure effect between the target system levels, established a target system effect analysis model, and gave a heuristic algorithm based on deep search to find key actions. Although the modeling method in the study can reduce the complexity of modeling the influence relationship in the target system, the cost of selecting key actions is not included in the evaluation of the effect of the target system. Qin et al., Li et al., and Yuan et al. [15–17] used methods such as fault tree or graph theory to describe the target system, but the uncertain factors of action results are not considered in these schemes.

Based on the complex network model constructed in this study, first, the degree of nodes is defined from two aspects, namely, the value of the node itself and the network value of the node. Regarding the composition of the value of the node itself, this study establishes a model of the relationship between the target and the war, the model of the importance of the target in the system, and the model of the threat of the target, which are used as the judgment scale of the value of the node. Regarding the network value of nodes, this study uses potential field theory and graph theory to describe the expansion degree based on the consideration of multiple influence factors between nodes. Second, using the advantages of the complex network model, this study adds the influence of the target cascade failure. The damage or loss of a node's function in the system network not only affects neighboring nodes but also indirectly affects multiple nodes that are not directly adjacent to it. The node degree and the effect of node failure together constitute the criterion to describe the network capability of the target combat system. Finally, this study uses the degree of decline in the network capability of the target combat system to measure the impact of the damage or loss of a node or multiple nodes and constructs a cost-effective function based on maximum entropy principle considering the cost of combat to select key targets weapons.

The rest of the study is organized as follows: Section 2 describes the construction of the complex network of the target combat system, Section 3 describes the construction of the key target selection model, Section 3.1 provides the target network system combat capability model mainly describing the definition and modeling of the node degree.  Section 3.2 provides the target network system cascade failure model mainly describing the direct and indirect influence degree and modeling of the node.  Section 3.3 provides the evaluation criterion function model mainly describing the constructed objective function, which is used to screen the final selected objective.  Section 4 is the case scenario and simulation analysis, and Section 5 is the conclusion.

## 2. Target Combat System Network Construction

The key to using complex network theory to describe the target combat system lies in the definition of nodes and edges in the network. The target combat system refers to an organic whole that is operated by various target systems in accordance with certain organizational relationships and can achieve combat missions. According to the functional characteristics of the target system, the target system can be divided into the reconnaissance and early warning system, command and control system, fire strike system, air defence and antimissile system, and integrated support system. Each target system is composed of multiple targets with corresponding functions and there exist command, coordination, and support relationship among different functional target units. Each target is abstracted as a node *v* of a complex network, and the relationship between a target and a target is abstracted as an edge *e* of the complex network. The target network system constructed can be represented by a graph model *G*(*V*, *E*). Define the node set as

(1) $$\begin{array}{c} V=\left\{v_{11},v_{12},\ldots v_{ij}\ldots ,v_{mn}\right\},\;i=1,2\ldots m;j=1,2\ldots n, \end{array}$$

where *i* is the number of systems included in the system network, and *j* is the number of target functional units included in each system in the system network.

Define the edge set as

(2) $$\begin{array}{c} E=\left\{e_{11},e_{12},\ldots e_{lk}\ldots ,e_{mn}\right\},\;l=1,2\ldots m;k=1,2\ldots n, \end{array}$$

where *l* is the relationship between different systems in the system network, and *k* is the number of target units which are related to the system.

Taking the target combat system network constructed shown in Figure 1 as an example, in the expression of the graph model *G*(*V*, *E*), the node set *V* is

(3) $$\begin{array}{c} V=\left\{v_{11},v_{12},\ldots v_{ij}\ldots ,v_{mn}\right\},\;i=1,2\ldots m;j=1,2\ldots n, \end{array}$$

where

(4) $$\begin{array}{c} i=\left\{\begin{array}{cc} 1\text{,} & \text{reconnaissance early warning system,}\\ 2, & \text{comprehensive support system,}\\ 3, & \text{command and control system,}\\ 4, & \text{fire strike system,}\\ 5, & \text{air defense and antimissile system,} \end{array}\right.\\ j=\left\{\begin{array}{cc} 6, & \text{number of units included in system }1\text{,}\\ 5, & \text{number of units included in system }2\text{,}\\ 7, & \text{number of units included in system }3\text{,}\\ 6, & \text{number of units included in system }4\text{,}\\ 6, & \text{number of units included in system }5\text{.} \end{array}\right) \end{array}$$

The edge set *E* is

(5) $$\begin{array}{c} E=\left\{e_{11},e_{12},\ldots e_{lk}\ldots ,e_{mn}\right\},\;l=1,2\ldots m;k=1,2\ldots n, \end{array}$$

where

(6) $$\begin{array}{c} l=\left\{\begin{array}{cc} 1, & \text{notification relations related to system }1\text{,}\\ 2, & \text{support relations related to system }2\text{,}\\ 3, & \text{command relations related to system }3\text{,}\\ 4, & \text{protection relations related to system }5\text{,} \end{array}\right.\\ k=\left\{\begin{array}{cc} 5, & \text{target units, related to system }1\text{,}\\ 4, & \text{target units, related to system }2,\\ 10, & \text{target units, related to system }3\text{,}\\ 4, & \text{target units, related to system }5\text{.} \end{array}\right) \end{array}$$

In some special situation, there are backup target units in some systems. We define this backup relationship as

(7) $$\begin{array}{c} E_{\text{extra}}=\left\{e_{1\text{extra}},e_{2\text{extra}},e_{3\text{extra}},e_{4\text{extra}},e_{5\text{extra}}\right\}, \end{array}$$

where

(8) $$\begin{array}{c} \left\{\begin{array}{c} e_{1\text{ extra}}=2,\text{ two backup relations in system }1\text{,}\\ e_{2\text{ extra}}=1,\text{ one backup relations in system }2\text{,}\\ e_{3\text{ extra}}=3,\text{ three backup relations in system }3\text{,}\\ e_{4\text{ extra}}=2,\text{ two backup relations in system }4\text{,}\\ e_{5\text{ extra}}=2,\text{ two backup relations in system }5\text{.} \end{array}\right) \end{array}$$

It should be noted that the combat system network shown in Figure 1 is an idealized distribution of combat functional units. Functional units with the same combat attributes are distributed in adjacent locations to form an enhanced functional system. In actual combat, the same type of functional units are often distributed in different locations and in different systems to support the normal operation of other combat units, that is, the same type of functional units in each system are allocated to form a complete combat unit with other different functional units. In the actual application of this model, cluster analysis is needed to reorganize and convert different functional units into the system network structure shown in Figure 1 in the study.

## 3. Key Target Selection Model

The key target selection model is mainly composed of three parts, namely, the target network system combat capability model, the target system cascade failure model, and the evaluation criterion function model.

### 3.1. Combat Capability Model of the Target Network System

It can be seen from the graph model *G*(*V*, *E*) shown in Figure 1 that the combat capability of the target system is mainly measured by the value of the node. The value of a node includes two aspects, one is the value of the node itself and the other is the network value of the node. The value of the node itself reflects the combat capability of each target unit, and the network value of the node reflects the cooperation ability between the target units. The cooperation ability may be formed by the cooperation of two target units or the cooperation of multiple target units. In this study, we consider that the collaboration capabilities of multiple target units are the sum of the pairwise collaboration capabilities of the corresponding target units. Then, the combat capability of the target system can be expressed as

(9) $$\begin{array}{c} F=F_{i}+F_{ij}, \end{array}$$

where *F*_*i*_ represents the combat capability of the *i*th target unit, and *F*_*ij*_ represents the collaboration capabilities between the *i*th target and the *j*th target.

For each node *V*={*v*_11_, *v*_12_,…*v*_*ij*_ …, *v*_*mn*_} in the target system network *G*(*V*, *E*), we assume its own value is *P*={*p*_11_, *p*_12_,…*p*_*ij*_ …, *p*_*mn*_}. The value of the node itself is composed of three factors, which are the degree of connection between the target and the war, the degree of importance of the target in the system, and the degree of threat of the target.

Assuming that the degree of connection between the target and the war is *R*, then

(10) $$\begin{array}{c} R=w_{\inf}C_{\inf}+w_{\text{air}}C_{\text{air}}+w_{\text{sea}}C_{\text{sea}},\\ \text{s.t}.\left\{\begin{array}{c} 0\leq C_{\inf},C_{\text{air}},C_{\text{sea}}\leq 1,\\ w_{\inf}+w_{\text{air}}+w_{\text{sea}}=1, \end{array}\right) \end{array}$$

where *C*_inf_, *C*_air_, *C*_sea_ are the values of the target associated with the seizure of information rights, air supremacy, and sea supremacy, and *w*_inf_, *w*_air_, *w*_sea_ are the weights.

Assuming that the degree of importance of the target in the system is *I*, then

(11) $$\begin{array}{c} I=\frac{D_{kj}\sum_{i=1}^{K}e_{ij}}{\sum_{k=1}^{K}\left(P_{kj}\sum_{i=1}^{K}e_{ij}\right)}, \end{array}$$

where *D*_*kj*_ is the connection degree of the node *j* in the system where the node is located in the target system network, and *e*_*ij*_ is the edge of the network graph model, representing various connection relations; if there is a direct collaboration relationship between the two target units, then 0 < *e*_*ij*_ ≤ 1, vice versa *e*_*ij*_=0.

Assuming that the degree of threat of the target is *T*, then

(12) $$\begin{array}{c} T=\sum_{k=1}^{N}\sum_{i=1}^{M}w_{k}v_{ki}A_{kij},\;0<A_{kij}\leq 1,\\ \begin{array}{cc} \text{s.t}. & \left\{\begin{array}{c} \sum_{k=1}^{N}w_{k}=1,\\ \sum_{i=1}^{M}v_{ki}=1, \end{array}\right) \end{array} \end{array}$$

where *A*_*kij*_ is the degree of influence of the *j*th target on the *i*th key action of the *k*th stage, *v*_*ki*_ is the weight coefficient of the *i*th key action of the *k*th stage, and *w*_*k*_ is the weight coefficient of the *k*th stage in all stages.

The final value of the node itself is

(13) $$\begin{array}{c} P=R+I+T. \end{array}$$

It should be noted that the calculation results of the three factors that make up the value of the node itself are of different orders of magnitude, and we uniformly standardize them within the range [0, 10].

We introduce potential field theory to express the network value of each node in the target combat system network *G*(*V*, *E*). Potential field theory is a theory put forward by British physicist Faraday to describe the interaction of objects. For any mass point in space, there is an action field around it, and the mass points in the action field will be affected by the field. Every object in the action field has an effect on other objects, and the potential function of its action is

(14) $$\begin{array}{c} \varphi_{i}=m_{i}\cdot \;\exp\left(-\frac{{\left\|x_{i}-x_{j}\right\|}^{2}}{\sigma^{2}}\right), \end{array}$$

where *m*_*i*_ represents the mass of object *i*, ‖*x*_*i*_ − *x*_*j*_‖ represents the distance between object *i* and object *j*, and *σ* represents the impact factor, normally *σ*=2.

There is an action field around each node in the target combat system network *G*(*V*, *E*), so a topological potential field is formed in the entire target system network [7], for ∀*v*_*j*_ ∈ *V*, the potential energy of *v*_*j*_ in the field of *v*_*i*_ is

(15) $$\begin{array}{c} \varphi_{v_{i}}\left(v_{j}\right)=p_{i}p_{j}\cdot \;\exp\left(-\frac{{\left\|v_{i}-v_{j}\right\|}^{2}}{\sigma^{2}}\right), \end{array}$$

where ‖*v*_*i*_ − *v*_*j*_‖ represents the distance between node *v*_*i*_ and *v*_*j*_. The position of the node is the latitude and longitude of the combat unit which it represents in the actual system.

Since the enemy target system network contains multiple nodes (target units), each node works together to form the topological potential field of the target system. The potential at the node *v* in the topological potential field is

(16) $$\begin{array}{c} \varphi \left(v\right)=\sum_{i=1}^{n}p_{i}\cdot \;\exp\left(-\frac{{\left\|v-v_{i}\right\|}^{2}}{\sigma^{2}}\right). \end{array}$$

In the topological potential field of the target system, *d*_*ij*_=‖*v*_*i*_ − *v*_*j*_‖ represents the shortest path distance between node *v*_*i*_ and *v*_*j*_, so for ∀*v*_*j*_ ∈ *V*, in the topological potential field, the topological potential energy [8] *φ*(*v*_*i*_) is

(17) $$\begin{array}{c} \varphi \left(v_{i}\right)=p_{i}\sum_{\begin{array}{c} j=1\\ j\neq i \end{array}}^{n}p_{j}\cdot \;\exp\left(-\frac{d_{ij}^{2}}{\sigma^{2}}\right). \end{array}$$

Considering the cooperative relationship between the target units, the combat capability of the target system can be expressed as

(18) $$\begin{array}{c} F=\sum_{i=1}^{n}\lambda_{i}p_{i}+\sum_{i=1}^{n}\left(\varphi \left(v_{i}\right)\cdot e_{ij}\right), \end{array}$$

where *λ*_*i*_ represents the importance degree of the *i*th target unit in the target system, and *p*_*i*_ represents the combat capability of the *i*th target unit. *p*_*i*_ and the collaboration degree *e*_*ij*_ between the target units is given by the expert scoring method.

Because the position of the target unit in the target network system is different, that is, the node position is different and its importance is also different, so *λ*_*i*_ can be expressed as the first-level expansion degree [7] of node *v*_*i*_:

(19) $$\begin{array}{c} \lambda_{i}=\frac{1}{d_{i}^{2}}\left(d_{i}+\sum_{k=1}^{d_{i}}D_{k}\right), \end{array}$$

where *d*_*i*_ represents the number of adjacent nodes of node *v*_*i*_, and *D*_*k*_ represents the number of adjacent nodes of the *k*th adjacent node of node *v*_*i*_.

### 3.2. Target System Cascading Failure Model

Due to the relationship of command and control, coordination, and support between target units, when one or more target units in the target system are destroyed, it may cause cascading failures of other target units. We define a triple Struct(*F*, *S*, *K*) to describe the cascading failure relationship [18–21] of the target system network, as shown in Figure 2.

*F*={*f*_1_,…, *f*_*i*_,…, *f*_*n*_} represents the set of combat operations result. *f*_*i*_ ∈ {0,1} represents whether the *i*th target unit (node) is hit. When *f*_*i*_=0, it means that the *i*th target unit (node) is not hit. When *f*_*i*_=1, it means that the *i*th target unit (node) is hit.

*S*={*s*_1_,…, *s*_*i*_,…, *s*_*n*_} represents the set of target unit state. *s*_*i*_ ∈ {0,1} represents the state of the *i* th target unit (node). When *s*_*i*_=0, it means that the *i*th target unit (node) is destroyed. When *s*_*i*_=1, it means that the *i*th target unit (node) is in normal operation.

*K*={*k*_*i*_}(1 ≤ *i* ≤ *n*) represents the set of the failure effects relationship between the target units. *k*_*i*_ ∈ {0,1} represents the impact of the failure of the neighboring node *s*_1_,…, *s*_*j*_,…, *s*_*k*_(1 ≤ *j* ≤ *k* < *n*) of the node *s*_*i*_ on the function of node *s*_*i*_. *k*_*i*_=0 is a logical “or” relationship, which refers to the succession or backup relationship between two nodes. *k*_*i*_=1 is the logical “and” relationship, which refers to the command, support, protection, notification, and coordination relationship between two nodes.

*s*_*j*_ pointing to *s*_*i*_ means that the failure of the *j*th target unit will cause the *i*th target unit to fail. *d*_*i*_ pointing to *s*_*i*_ means that the *i*th target unit is destroyed by a strike action, so

(20) $$\begin{array}{c} s_{i}=\left\{\begin{array}{cc} 0, & f_{i}=1,\\ \prod_{j=1}^{k}\left|s_{j}\right|, & f_{i}=0,k_{i}=1,\\ 1-\prod_{j=1}^{k}\left(1-\left|s_{j}\right|\right), & f_{i}=0,k_{i}=0. \end{array}\right) \end{array}$$

### 3.3. Evaluation Criterion Function Model

Medium and long-range conventional weapon fire strikes are used to strike the enemy's strategic targets, such as airports and large hydropower stations, to interfere with the enemy's normal life and disrupt the logistics support of combatants or directly attack the enemy's combat forces so that the enemy's combat capabilities cannot be used, thus ensuring our safety. The effectiveness of medium and long-range conventional weapons firepower is usually measured by the decline in the enemy's combat capability. Modern warfare is fast-paced, and the conventional combat idea is to select key targets in the enemy's target system to give key firepower strikes, creating a chain reaction of damage, and making the enemy's overall combat capability drop in an “avalanche” manner, so as to break the network and the chain and achieve the effect of destroying a point like destroying a plane [22–32].

Assuming that the initial combat capability of the enemy's target system is *F*_0_, after the cost of firepower *x*_1_ is used to strike the enemy's *x*_2_ targets, the combat capability of the enemy's target system is *F*_1_, and then, the reduction in the combat capability of the target system is

(21) $$\begin{array}{c} \Delta F_{x}=F_{0}-F_{1}=F_{x}+F_{x\_\text{out}}+F_{x\_\text{enter}}, \end{array}$$

where *F*_*x*_ represents the sum of combat capabilities of *x*_2_ targets, *F*_*x*_out_ represents the sum of topological potential energy of *x*_2_ targets, namely, the cascading failure effect, and *F*_*x*_enter_ represents the sum of topological potential energy of *x*_2_ targets affected by other targets, namely, the collaboration capabilities between targets.

Since there are *C*_*n*_^*x*^ schemes when selecting *x* targets from *n* targets for fire strike, then one scheme that maximizes the reduction in the overall combat capability of the target system can be selected through sequencing, namely, maxΔ*F*_*x*_.

Taking into account the principle of optimal efficiency-cost ratio and maximum entropy theory, the evaluation criterion function model is

(22) $$\begin{array}{c} \left\{\begin{array}{c} f=\max\left(\frac{\max\Delta F_{x}}{x_{1}x_{2}}\right),\\ \begin{array}{cc} \text{s.t.} & 1\leq x_{2}\leq n. \end{array} \end{array}\right) \end{array}$$

## 4. Case Analysis

### 4.1. Basic Scene

Assume that the enemy's combat system is a network consisting of 25 targets in 5 types of target systems, as shown in Figure 3. The combat capabilities of various target units are obtained based on the constructed node degree model and expert suggestions. The degree of collaboration between target units is scored by experts, as given in Tables 1 and 2, respectively.

### 4.2. Simulation Calculation

According to the key target selection model, the value of each node itself, the network value of each node, and the cascading failure impact ability of each node (target unit) in the target combat system network can be got by using MATLAB, and the simulation results are given in Table 3.

Through MATLAB simulation, the combat capability decline value of the target system and the selected key targets can be obtained as given in Table 4.

It can be seen from Table 4 that when striking three targets, the maximum efficiency-cost ratio is 117.2873. The key targets are air defence position 5, air defence position 1, and satellite reception center 1. The screening results of the key targets are also in line with the actual combat situation. The three key targets selected first have the characteristics of complex nodes and occupy an important position in the network. Second, there are no weapon positions among the key targets screened, which means that although the network considers that weapon positions are important, striking a few weapon positions has little effect on the combat capability of the entire target combat system network because there are many other weapon positions playing the same role. Finally, the key targets selected are the protection layer and communication center of the target combat system network. In actual operations, it is equivalent to blinding the vision and hearing of the enemy's target combat system and making it extremely easy to attack. In summary, the above screening results are reasonable and can play a supporting role in combat.

Compared with other methods, this key target selection method considers many factors and is complicated, which is very in line with the complex situation of information warfare system confrontation, and can provide good suggestions for commanders' decision-making.

## 5. Conclusion

Based on the complex network theory, this study constructs the target combat system network and comprehensively establishes the node degree value model, the cascade failure model, and the evaluation criterion function model to assist the commander in the selection of key targets. This method intuitively demonstrates the complexity of the system's network confrontation, simulates the complex battlefield factors in a deeper level, and plays a good auxiliary role for the commander to choose the target of the medium and long-range conventional weapons. The next step in this study is to optimize the constructed complex network model, further model the cost of weapon consumption in the evaluation criterion function, and consider adding the cost of strike risk instead of a single index of the number of medium and long-range conventional weapons.

## Figures and Tables

**Figure 1:** Target combat system network.

**Figure 2:** Target cascading failure relationship.

**Figure 3:** The enemy target system figure in assumption.

**Table 1:** Various target combat capabilities.

Name	Combat capability
Command post	7
Radar station	3
Satellite reception center	4
Weapon position	6
Air defence position	5
Airport	4
Comprehensive support warehouse	4

**Table 2:** Collaboration degrees between targets.

Collaboration relationship	Collaboration degree
Command	0.3
Notification	0.2
Protection	0.2
Support	0.2
Backup	0.1

**Table 3:** Related data for each target.

Number	Target *i*	Combat capability *F*_*i*_		Topological potential energy *φ*(*v*_*i*_)	The potential energy of other targets against target *iφ*′(*v*_*i*_)
1	Command post 1	11.4800	17.5567		33.8143
2	Command post 2	4.1481	6.6685		34.1754
3	Command post 3	3.7100	22.4480		36.7187
4	Command post 4	5.6389	4.4411		25.15423
5	Satellite reception center 1	4.0000	57.3273		13.1153
6	Satellite reception center 2	3.7778	2.5294		12.9162
7	Radar station 1	4.6875	20.9707		9.0189
8	Radar station 2	3.0000	27.1355		8.4718
9	Air defence position 1	4.0278	78.7594		20.5700
10	Air defence position 2	7.8125	13.7948		16.7233
11	Air defence position 3	5.0000	19.7929		17.0897
12	Air defence position 4	3.4000	6.1607		11.8701
13	Air defence position 5	6.8750	81.3892		15.7980
14	Weapon position 1	9.0000	21.4847		30.0457
15	Weapon position 2	9.0000	6.0908		37.0893
16	Weapon position 3	9.0000	22.4092		36.4239
17	Weapon position 4	9.0000	6.7095		27.7353
18	Weapon position 5	9.0000	1.4248		35.8225
19	Weapon position 6	9.0000	1.1046		27.7778
20	Airport 1	4.0000	20.4119		18.1016
21	Airport 2	12.0000	12.7517		16.5835
22	Airport 3	12.0000	48.8900		20.3458
23	Comprehensive support warehouse 1	3.3600	28.5714		11.3143
24	Comprehensive support warehouse 2	4.4800	18.9048		15.9266
25	Comprehensive support warehouse 3	2.6939	4.3302		12.1777

**Table 4:** The combat capability decline value of the target system and the selected key targets.

Overall cost *x*_1_*x*_2_	Decline value of combat capability maxΔ*F*_*x*_	Efficiency-cost ratio maxΔ*F*_*x*_/*x*_1_*x*_2_	Selected targets *i*
1	104.0622	104.0622	Air defence position 5

2	231.4194	115.7097	Air defence position 5
			Air defence position 1

3	351.8620	117.2873	Air defence position 5
			Air defence position 1
			Satellite reception center 1

4	420.0978	105.0245	Air defence position 5
			Air defence position 1
			Satellite reception center 1
			Airport 3

5	492.9309	98.5862	Air defence position 5
			Air defence position 1
			Satellite reception center 1
			Airport 3
			Weapon position 3

## Data Availability

The dataset used to support this study is available from the corresponding author upon request.
